The article "Acupuncture for Vascular Dementia: A Pragmatic Randomized Clinical Trial" was published in 2015. Journal: ScientificWorldJournal.

# Acupuncture for Vascular Dementia: A Pragmatic Randomized Clinical Trial

**DOI:** 10.1155/2015/161439

**Published:** 2015-10-01

**Authors:** Guang-Xia Shi, Qian-Qian Li, Bo-Feng Yang, Yan Liu, Li-Ping Guan, Meng-Meng Wu, Lin-Peng Wang, Cun-Zhi Liu

**Affiliations:** ^1^Acupuncture and Moxibustion Department, Beijing Hospital of Traditional Chinese Medicine Affiliated to Capital Medical University, 23 Meishuguanhou Street, Dongcheng District, Beijing 100010, China; ^2^Acupuncture and Moxibustion Research Institute, The First Hospital Affiliated to Tianjin College of Traditional Chinese Medicine, 314 West Anshan Avenue, Tianjin 300193, China

## Abstract

In this trial, patients who agreed to random assignment were allocated to a randomized acupuncture group (R-acupuncture group) or control group. Those who declined randomization were assigned to a nonrandomized acupuncture group (NR-acupuncture group). Patients in the R-acupuncture group and NR-acupuncture group received up to 21 acupuncture sessions during a period of 6 weeks plus routine care, while the control group received routine care alone. Cognitive function, activities of daily living, and quality of life were assessed by mini-mental state examination (MMSE), Activities of Daily Living Scale (ADL), and dementia quality of life questionnaire (DEMQOL), respectively. All the data were collected at baseline, after 6-week treatment, and after 4-week follow-up. No significant differences of MMSE scores were observed among the three groups but pooled-acupuncture group had significant higher score than control group. Compared to control group, ADL score significantly decreased in NR-acupuncture group and pooled-acupuncture group. For DEMQOL scores, no significant differences were observed among the three groups, as well as between pooled-acupuncture group and control group. Additional acupuncture to routine care may have beneficial effects on the improvements of cognitive status and activities of daily living but have limited efficacy on health-related quality of life in VaD patients.

## 1. Introduction

Vascular dementia (VaD) is thought to be resulted from various types of ischemic and hemorrhagic brain lesions which lead to intellectual and physical disability [1]. It is the second most common cause of dementia among the older people, representing 15–25% of all cases worldwide [2–4]. Projections indicate that progressive ageing of the populations and the high prevalence of cerebrovascular and cardiovascular pathologies capable of producing VaD are the most common form of dementia [5, 6]. This creates a difficult situation for those suffering from VaD, their caregivers, and healthcare providers. However, definitive medical or surgical treatments do not exist so far [7, 8].

The article "Acupuncture for Vascular Dementia: A Pragmatic Randomized Clinical Trial" was published in 2015. Journal: ScientificWorldJournal.

Maintaining or improving quality of life in people with VaD is currently a key outcome of health services and the increasing number of psychosocial interventions targeting this population [9]. Being not able to perform basic activities of daily living reduces quality of life in dementia [10], including bathing, continence, dressing, feeding, toileting, and transfer. Since the need for assistance in these activities makes people with VaD dependent on informal (family) or formal (professional) care, quality of life is one of the most important outcomes in improving well-being of people with VaD [11, 12].

Acupuncture is a core component in traditional Chinese medicine (TCM) and can be traced back more than 3000 years in China. It is often used as a treatment for dementia [13, 14]. Nevertheless, recent systematic review has shown inconclusive evidence because of low methodological quality [13]. The effectiveness of acupuncture for VaD has not been fully established. The majority of previous trials for acupuncture were designed for experimental studies [15]. Hence, there is currently very little information about the effectiveness of acupuncture in general medical practice.

Based on our previous study [16], we designed the present study as a pragmatic trial to investigate the effectiveness of acupuncture in addition to routine care among patients with VaD. In addition, we examined whether the effects of acupuncture differ between randomized and nonrandomized patients.

## 2. Experimental

### 2.1. Methods

Patients were eligible for this trial only after they had met rigorous criteria for probable VaD as defined by the National Institute of Neurological Disorders and Stroke-AIREN criteria (NINDS-AIREN). Inclusion criteria also included a score of 0 to 23 on the mini-mental state examination (MMSE), disease duration of more than 2 months, onset of the disease at age less than 80 years, and the availability of a reliable caregiver. All subjects included in the trial were evaluated with the Hachinski Ischemic Score (HIS). A HIS of ⩾7 has been validated in an autopsy study as an accurate indicator of VaD [17]. Participants were excluded if they had a prior diagnosis of Alzheimer's disease (AD), Parkinson disease, Huntington disease, and other neurodegenerative dementia. Participants with less than secondary education were ineligible in the present study. Exclusion criteria also included the presence of abnormal executive control function, severe enough to interfere with social or occupational functioning and inability to give consent because of impaired cognition or receptive aphasia. All patients have undergone a neurologic interview to determine their history of onset, symptoms, and recovery from stroke in the first interview.

The article "Acupuncture for Vascular Dementia: A Pragmatic Randomized Clinical Trial" was published in 2015. Journal: ScientificWorldJournal.

We performed the study according to common guidelines for clinical trials (Declaration of Helsinki, International Conference on Harmonisation (ICH)/WHO Good Clinical Practice standards (GCP) including certification by an external audit). The trial protocol has been approved by the Research Ethical Committee of The First Hospital affiliated to Tianjin College of Traditional Chinese Medicine (20073055). All study participants provided written, informed consent.

### 2.2. Randomization

Patients who agreed to be randomly assigned were allocated to a randomized acupuncture group (R-acupuncture group) or control group. Block randomization with a block size of 4 was by sequential, sealed, opaque envelopes. It occurred after the acupuncturist's evaluation (concealed allocation) using a computer-generated, random-allocation sequence (random list generated with SAS 8.2). Furthermore, participants who did not consent to randomization were assigned to a nonrandomized acupuncture group (NR-acupuncture group). We ensured that the patients, data collection staff, and data analysts were blinded during the study period; they were all unaware of the randomization. The acupuncturists were not blinded to the treatments they delivered because acupuncture manipulation made this impossible. During the intervention, acupuncturist and the personnel who collected data were segregated by an opaque screen immediately after the treatment started and were instructed not to exchange information with each other.

### 2.3. Intervention

Patients in the R-acupuncture group and NR-acupuncture group received acupuncture treatment plus routine care, while those in the control group received routine care alone. Routine care here refers to the use of certain medications. These medicines include antiplatelet agents (aspirin or ticlopidine), antihypertensive, diuretics, and nimodipine and should be taken following the advice of physician. In addition, they received a weekly phone call to inquire of their health status to provide individual attention. Acupuncture was administrated by 5 therapists with more than 6 years of experience and a Chinese medicine practitioner license from the Ministry of Health of the People's Republic of China. Based on the TCM theory, the main acupoints we selected were as follows: GV20 (baihui), EX-HN1 (sishencong), GV24 (shenting), CV17 (tanzhong), PC6 (neiguan), CV12 (zhongwan), CV6 (qihai), SP10 (xuehai), and ST36 (zusanli). Moreover, the following acupoints could be added as auxiliary acupoints: GB 20 (fengchi), ST40 (fenglong), LR3 (taichong), SP6 (sanyinjiao), and ST25 (tianshu). The acupuncture point prescriptions used were individualized to each patient and were at the discretion of the acupuncturist. Acupuncture was performed by means of standard stainless-steel needles (0.25 Φ  × 25 mm and 0.25 Φ  × 40 mm, Beijing Hanyi Medical Instrument Center) and manually stimulated to elicit needle sensation (de qi). The treatment consisted of 21 sessions of 30 minutes' duration, and each was administered once every other day over a period of 6 weeks.

The article "Acupuncture for Vascular Dementia: A Pragmatic Randomized Clinical Trial" was published in 2015. Journal: ScientificWorldJournal.

### 2.4. Measurements

Demographic measures collected at the baseline evaluation included age, gender, common complications of VaD, HIS, and outcome variables.

Cognitive status, including orientation, memory, calculation, language, and constructional apraxia, of the VaD patients was assessed using the MMSE. Total scores for this measure range from 0 to 30, with lower scores indicating lower cognitive functioning.

Activities of daily living were determined by Activity of Daily Living Scales (ADL). It has been developed specifically for use with VaD, consisting of 20 daily-living abilities, where higher scores indicate lower levels of activities of daily living (scores range from 0 to 60).

Health-related quality of life is measured by dementia quality of life questionnaire (DEMQOL). It is a tool with which to evaluate whether the interventions and services achieve this. It covers five domains of quality of life and uses both self-reporting and rating by family guardian or staff member as proxy. Higher scores indicate better quality of life and vice versa. It has good internal consistency, interior reliability, and concurrent validity and can generate a measure of utility.

All the outcomes were assessed at baseline, after 6-week treatment and after 4-week follow-up.

### 2.5. Sample Size Calculation

According to previous study, there was a significant difference between the pre- and post-treatment for the treatment group than that for the control group with an increase of 4.27 ± 2.05. We calculated the number of sample size, using the following formula:

(1) n1=n2=2tα+tβsδ2(α=0.05, β=0.10) δ=1.84, s=1.56.

As a result, we estimated that 20 patients were required in each group. Assuming a 20% drop-out rate, we planned to randomize 24 patients to each arm.

### 2.6. Statistical Analysis

A per protocol analysis was done based on patients with no major protocol violations by the end of 4-week follow-up after randomization. Data are expressed as mean ± standard deviation (SD), or frequencies and percentages, according to the type of variable. For the between-group comparisons at baseline, either the Chi-Square test or one-way ANOVA was used. An analysis of covariance with additional covariate of age was performed to account for potential baseline differences. Repeated-measures analysis of variance was used to determine whether significant differences exist across time. Furthermore, results were evaluated by pooling all patients who received acupuncture treatment into one group. Pooled-acupuncture group which actually contained patients in R-acupuncture group and NR-acupuncture group were compared with the control group. *P* values lower than 0.05 were considered to be statistically significant. Statistical analysis was performed with SPSS version 10.0 (SPSS Inc., Chicago, Illinois, USA).

The article "Acupuncture for Vascular Dementia: A Pragmatic Randomized Clinical Trial" was published in 2015. Journal: ScientificWorldJournal.

## 3. Result

### 3.1. Patient Enrollment

In the present population-based study, patients managed in the community as well as those managed in hospital (Tianjin, china) were recruited from June 2007 to February 2010.  Figure 1 showed the flow of participants through the trial. Of 120 screened patients, 52 could not be included in the study, mainly because they did not meet all eligibility criteria. A total of 68 patients were included. Of these, 24 were randomly assigned to R-acupuncture and 24 to control group. 20 patients who declined randomization were allocated to NR-acupuncture group. Five patients dropped out during the trial, accounting for a 7.4% dropout rate. Among the 5 dropouts, 1 patient had recurrent stroke, 1 patient died because of heart attacks, 2 patients did not tolerate needling, and 1 patient withdrew due to move from one city to another. Thus, the protocol analysis included 63 patients.

### 3.2. Analysis of Baseline Data

The demographic and clinical features at baseline are shown in Table 1. Three groups were comparable with regard to most baseline characteristics except for age. Patients in the randomization group were, on average, younger than those in the other two groups (*P* = 0.003).

### 3.3. Analysis of Outcome Variables

Repeated-measures analysis of variance on MMSE scores revealed a time effect (*P* = 0.034) and a treatment × time interaction (*P* = 0.001), indicating a favorable improvement in the cognitive evolution of VaD individuals as the extension of time (Figure 2(a)). No significant differences of MMSE were observed among the three groups. However, pooled-acupuncture group had significant higher score than control group (*P* = 0.014) (Figure 2(b)).

Figure 3(a) indicated no time effect (*P* = 0.241), but a treatment effect (*P* = 0.027) and treatment × time interaction (*P* = 0.014) on ADL score. Lower score was observed in the NR-acupuncture group compared to the control group (*P* = 0.01). Nonetheless, no significant differences were detected in R-acupuncture group versus NR-acupuncture group (*P* = 1.00), as well as R-acupuncture group versus control group (*P* = 0.067). In addition, lower score was found in pooled-acupuncture group compared to the control group (*P* = 0.003) (Figure 3(b)).

The article "Acupuncture for Vascular Dementia: A Pragmatic Randomized Clinical Trial" was published in 2015. Journal: ScientificWorldJournal.

Figure 4 showed a time effect (*P* = 0.000) and treatment × time interaction (*P* = 0.011) and no treatment effect (*P* = 0.05) on DEMQOL score, indicating a significant improvement on health-related quality of life across time. However, no significant differences were observed among the three groups (Figure 4(a)). Besides, no significant differences existed between the pooled-acupuncture group and control group (*P* = 0.283) (Figure 4(b)).

### 3.4. Safety of Acupuncture

During the acupuncture treatment, 25% experienced discomfort at the sites of needle insertion or simulated needle insertion, and 20% had bruising. No serious adverse events were documented.

## 4. Discussion

The aim of our study was to examine whether acupuncture has additional value in patients with VaD compared to treatment with routine care alone. Results indicate that, compared to patients in control group, those in pooled-acupuncture group showed significant improvements in cognitive status and activities of daily living. Moreover, patients who declined randomization and therapeutic outcomes after acupuncture were better than those who consented to. Additional acupuncture to routine care is of limited efficacy in VaD patients whose health-related quality of life has already deteriorated.

Recent international policy guidelines aim to promote independence in dementia and show a rising interest in how nonpharmacological interventions could help maintain everyday functional independence as long as possible [18]. This information could contribute to shaping interventions to help VaD remain at home as long as possible and maintain a good health-related quality of life.

There is growing evidence implicating dementia is a risk factor for stroke and stroke is associated with an increased risk of subsequent dementia [2, 19, 20]. Although most stroke survivors go on to show some improvement over time, a large percentage eventually develops significant symptoms of dementia [21, 22]. Acupuncture is frequently advocated as an adjunct treatment during stroke rehabilitation. However, controversy remains regarding the effectiveness of acupuncture for recovery in activities of daily living and health-related quality of life after stroke [19, 23]. A recent meta-analysis of data from rigorous randomized sham-controlled trials did not show a positive effect of acupuncture as a treatment for functional recovery after stroke [14]. Park et al. [24] reported that acupuncture is not superior to sham treatment. Nonetheless, Moffet [25] argued that even if acupuncture is ineffective for stroke itself, it may nonetheless be helpful in treating pain, sleep disturbance, anxiety, depression, or other conditions that are common consequence of stroke and that are often barriers to rehabilitation and recovery. Kwok et al. [26] showed that acupuncture elicited significant improvement in sleep quality of elders with dementia in terms of significant gain in resting time as well as sleep time in the treatment period over the control period. Preliminary searches revealed more than 105 studies of acupuncture for treating vascular dementia. Benefit was reported in up to 70 to 91% of the treatment group. However, one review in 2007 suggested there is currently no evidence available from sufficiently high quality randomized controlled trials to allow assessment of the efficacy of acupuncture in the treatment of vascular dementia [27]. Our results showed a beneficial effect of additional acupuncture on cognitive status and activities of daily living for VaD patients.

The article "Acupuncture for Vascular Dementia: A Pragmatic Randomized Clinical Trial" was published in 2015. Journal: ScientificWorldJournal.

We took a pragmatic approach, aiming to evaluate acupuncture in a manner that would reflect as closely as possible the conditions of daily medical practice. The additional inclusion of patients who declined randomization allowed us to investigate any potential selection effects. One explanation for the significant improvements in NR-acupuncture group may attribute to potent placebo effects. Previous studies have shown that expectancy, a crucial component of placebo, plays an important role in acupuncture treatment efficacy [28]. Linde et al. [29] suggested that expectancy is able to enhance acupuncture analgesia initiated by an inhibited brain response to calibrated pain stimuli. They showed strong association between better improvement and higher expectations by a pooled analysis of four randomized controlled trials of acupuncture in patients with chronic pain. Patients refusing randomization tend to believe that they were assuring to get an active or a more effective intervention. Hence, patient expectations may play a more prominent role than those of patients receiving randomization.

Treatment of VaD also includes prevention and attenuation of potential risk factors [4, 30]. There is evidence that the treatment of modifiable vascular risk factors, such as hypertension, diabetes mellitus, hypercholesterolemia, and heart disease, is likely to slow the progress of cognitive decline and a reduction of the risk of dementia [31, 32]. Park et al. indicating that the beneficial effect of acupuncture could be of clinical importance to prevent the progression of cardiovascular diseases [33]. The main finding in the present study was that additional acupuncture treatment was efficacious in reducing and controlling clinical syndrome associated with VaD. Therefore, future researches should provide answers regarding the beneficial effect of acupuncture on modifying risk factors of VaD.

The article "Acupuncture for Vascular Dementia: A Pragmatic Randomized Clinical Trial" was published in 2015. Journal: ScientificWorldJournal.

In a pragmatic trial, it is not usually appropriate to use a placebo control and blinding, as these are likely to have a detrimental effect on the trial's ecological validity [34]. So, we compared the effect of acupuncture with another treatment, not with a placebo and the sham acupuncture. Our study has some limitations. Firstly, the treatment time is relatively short. This study demonstrated that the 6-week treatment of acupuncture in VaD patients improves cognitive function and activities of daily living but did not change the health-related quality of life. The potential role of acupuncture treatment for long-term therapy has not been examined. Further studies will be necessary to demonstrate whether long-term acupuncture treatment can sustain the improvement. In addition, we consider that a longer period of follow-up could be necessary to investigate the optimum timing for such an acupuncture treatment and to assess the value of repeated courses of acupuncture for patients experiencing VaD. Secondly, because the recruitment was limited due to administrative factors, our results need to be further investigated in the future studies with larger number of patients. Another potential limitation is that whether acupuncture had an independent beneficial effect on VaD remains unexplained in the present trial.

## 5. Conclusion

Our study shows that additional acupuncture to routine care may have beneficial effects on the improvements of cognitive status and activities of daily living but have limited efficacy on health-related quality of life in VaD patients.

## Figures and Tables

**Figure 1:** Trial flow chart.

**Figure 2:** The changes of score in MMSE across time. Comparison among R-acupuncture group, NR-acupuncture group, and control group (a) and between pooled-acupuncture group and the control group (b). R-acupuncture = randomized acupuncture group, Control = control group, NR-acupuncture = nonrandomized acupuncture group, and P-acupuncture = pooled-acupuncture group. T1 = at baseline, T2 = after 6-week treatment, and T3 = after 4-week follow-up.

**Figure 3:** The changes of score in ADL across time. Comparison among R-acupuncture group, NR-acupuncture group, and control group (a) and between pooled-acupuncture group and the control group (b). R-acupuncture = randomized acupuncture group, Control = control group, NR-acupuncture = nonrandomized acupuncture group, P-acupuncture = pooled-acupuncture group. T1 = at baseline, T2 = after 6-week treatment, and T3 = after 4-week follow-up.

The article "Acupuncture for Vascular Dementia: A Pragmatic Randomized Clinical Trial" was published in 2015. Journal: ScientificWorldJournal.

**Figure 4:** The changes of score in DEMQOL across time. Comparison among R-acupuncture group, NR-acupuncture group, and control group (a) and between pooled-acupuncture group and the control group (b). R-acupuncture = randomized acupuncture group, Control = control group, NR-acupuncture = nonrandomized acupuncture group, and P-acupuncture = pooled-acupuncture group. T1 = at baseline, T2 = after 6-week treatment, and T3 = after 4-week follow-up.

**Table 1:** Subjects' baseline characteristics.

	R-acupuncture (*n* = 22)	NR-acupuncture (*n* = 19)	Control (*n* = 22)
Gender *n* (%)			
Men *n* (%)	12 (54.55)	6 (31.58)	11 (50.00)
Women *n* (%)	10 (45.45)	13 (68.42)	11 (50.00)
Age (M ± SD, y)	67.24 ± 9.33^*^	57.21 ± 10.80^*^	67.45 ± 10.14^*^
Hypertension, *n* (%)	17 (77.27)	17 (89.47)	15 (68.18)
Diabetes mellitus, *n* (%)	2 (9.10)	4 (21.05)	4 (18.18)
Coronary heart disease, *n* (%)	9 (40.91)	7 (36.84)	8 (36.37)
HIS (M ± SD)	9.55 ± 2.37	11.32 ± 2.16	11.00 ± 2.14
MMSE (M ± SD)	18.27 ± 4.08	17.74 ± 3.33	17.77 ± 3.99
ADL (M ± SD)	42.91 ± 13.97	43.84 ± 11.42	49.86 ± 14.97
DEMQOL (M ± SD)	72.41 ± 7.02	64.68 ± 6.68	72.27 ± 9.23

^*^Differences among the three groups are statistically significant *P* < 0.05. R-acupuncture = randomized acupuncture group; Control = control group; NR-acupuncture = nonrandomized acupuncture group; HIS = Hachinski Ischemic Score; MMSE = mini-mental state examination; ADL = activities of daily living; DEMQOL = health-related quality of life.

## Abbreviations

VaD: Vascular dementia
R-acupuncture group: Randomized acupuncture group
NR-acupuncture group: Nonrandomized acupuncture group
MMSE: Mini mental state examination
ADL: Ability of daily life scale
DEMQOL: Dementia quality of life questionnaire
TCM: Traditional Chinese medicine
HIS: Hachinski Ischemic Score
AD: Alzheimer's disease
SD: Standard deviation.
